The article "The Factors Affecting Orthodontic Pain with Periodontitis" was retracted in 2023. Reasons: suspected computer-generated content; unreliable results or conclusions; lack of ethics approval or compliance; missing or withdrawn patient consent.

# The Factors Affecting Orthodontic Pain with Periodontitis

**DOI:** 10.1155/2021/8942979

**Published:** 2021-11-01

**Authors:** Yuzhi Peng, Songjiang Tang

**Affiliations:** ^1^Department of Stomatology, First Affiliated Hospital of Guizhou University of Traditional Chinese Medicine, Guiyang 550001, China; ^2^Department of Anesthesiology, First Affiliated Hospital of Guizhou University of Traditional Chinese Medicine, Guiyang 550001, China

## Abstract

The occurrence of pain is often closely related to the psychological status, and the threshold for pain tolerance varies from patient to patient. In short, the factors affecting orthodontic pain are diverse and have individual differences. Tooth pain after the first force of intraoral malocclusion orthodontic treatment is one of the common complications of fixed orthodontic treatment, which often affects the outcome of treatment of patients with malocclusion and their subjective satisfaction with fixed orthodontic treatment. The purpose of the paper was to investigate the basic patterns and influencing factors of dental pain in fixed orthodontic patients within seven days after the initial wearing of straight arch aligners and the analysis of the effect of psychological intervention on dental pain using the visual simulation scoring method. According to the inclusion criteria of the experimental design, 89 patients who visited the Department of Orthodontics of Hospital for malocclusion were randomly divided into observation group and control group, and the observation group used chewing gum as psychological intervention, while the control group did not use any intervention. The effect of psychological intervention on periodontal pain was analyzed. The results of the paper were that all but 3 of the 89 patients had no pain, and all the patients had different degrees of dental pain at different points in time.

## 1. Introduction

With the development of society, the progress of technology, and the improvement of living conditions, people are no longer just satisfied with the level of subsistence but have higher and higher requirements for the quality of life and also have higher and higher requirements for aesthetics [1]. In order to make oneself more beautiful and confident, the treatment of maxillofacial deformities has entered people's vision and attracted widespread attention. In recent years, the prevalence of maxillofacial malocclusion in China has shown an increasing trend, and according to the latest research data, it can be as high as 72.92% [2]. Dental and maxillofacial malocclusion is a congenital or externally acquired abnormality in the morphology and structure of the teeth and jaws and the function of the accompanying oromandibular system, which has become one of the most important diseases threatening the physical and mental health of the nation, and the World Health Organization has positioned oral and maxillofacial malocclusion as one of the three major symptoms of oral diseases [3]. Malocclusion not only affects the physiological function of the oral cavity but also has an impact on other oral diseases such as endodontic disease and periodontal disease.

The article "The Factors Affecting Orthodontic Pain with Periodontitis" was retracted in 2023. Reasons: suspected computer-generated content; unreliable results or conclusions; lack of ethics approval or compliance; missing or withdrawn patient consent.

Nowadays, with the change of the medical model, the definition of health not only includes the physiological health of the human body but also the psychological perfection state [4]. The low-level goal is to restore and reconstruct the normal anatomical structure of the patient's maxillofacial tissues without affecting the patient's mastication, swallowing function and breathing, and other physiological functions and to achieve the maximum degree of aesthetics, while the high-level goal is to understand the psychological state of the patient and family as much as possible, help them overcome their psychological fears, and improve their self-confidence, so that they can get a higher degree of cooperation from the patient [5–8], thus ensuring that orthodontic treatment is carried out effectively and smoothly. Studies have been done on patients with malocclusion and have shown that orthodontic therapeutic pain not only affects patients with malocclusion in fixed orthodontic treatment but also causes patients with fixed orthodontic treatment to fail to attend follow-up appointments or even to terminate their orthodontic treatment, and other studies have shown that about eight percent of patients give up the pursuit of aesthetics because of the severe pain caused by orthodontic treatment [9].

Therefore, the pathogenesis of dental pain, its development, the factors influencing it, and the relief of orthodontic pain have always been of interest. The transmission of pain is analyzed biologically, the tooth is stimulated, capillaries in the pulp are dilated and filled with blood, the osmotic pressure in the pulp cavity is increased, plasma extravasation and microcirculatory disorders increased pressure in the pulp tissue, and conduction via C and A-*δ* nerve fibers in the pulp cavity induced tooth pain. After periodontal membrane stimulation, the periodontal ligament is compressed or stretched. Mast cells release various inflammatory factors and pain-causing substances. A series of edema and inflammatory reactions are as follows: vasodilatation and congestion, an increase in capillary osmotic pressure, an increase in sensitivity of receptors in the periodontal membrane, and a decrease in the body's threshold for dental pain response [10]. Early pain often occurs after the application of orthodontic forces, causing changes in the osmotic pressure in the periodontium; delayed pain is an allergic state of the periodontium, probably related to the stimulation of the nerve endings of the periodontium by inflammatory mediators, which in turn stimulates the release of neuropeptides from the pain receptors, usually within a few hours after the force is applied. The pain stimulus signals from the tooth and periodontal membrane continue to transmit pain stimulus signals to the center on the one hand and release neuropeptides (enkephalins, histamine, interleukins, substance P, dopamine, gamma-aminobutyric acid, serotonin, glycine, prostaglandins, calcitonin gene-related peptide CGRP, neurofilament protein NEP, vasoactive intestinal peptide, neuropeptide, etc.) to the periphery to regulate orthodontic pain, and these released neuropeptides are also involved in local blood flow regulation, which facilitates the reconstruction of dental tissue [11].

The article "The Factors Affecting Orthodontic Pain with Periodontitis" was retracted in 2023. Reasons: suspected computer-generated content; unreliable results or conclusions; lack of ethics approval or compliance; missing or withdrawn patient consent.

A person's psychological state can affect his or her perception of orthodontic pain during the treatment process, so psychological interventions can be used to improve patient cooperation, relieve orthodontic pain, ensure the smooth and effective implementation of orthodontic fixed orthodontic treatment, and improve patients' oral health-related quality of life under the modern biopsychosocial medicine model. Quality of life should be improved to find a simple, effective, easy-to-implement method with few side effects for orthodontic treatment pain relief and to provide some theoretical basis for psychological interventions affecting orthodontic dental pain. The purpose of this experiment is to investigate the changes in the pattern of dental pain, the factors affecting the pain, and the psychological intervention on dental pain within one week after the first force application of straight wire orthodontic appliances in patients with malocclusion by means of a clinical questionnaire, so as to provide a theoretical basis for the development of orthodontic clinical work.

## 2. Related Work

Over the years, the study of pain response to fixed orthodontic treatment has become a hot research topic in orthodontic medicine. Clinical research focuses on the manifestation of pain, influencing factors, and how to relieve the symptoms of pain, while basic research focuses on the causes, influencing factors, and pathogenesis of orthodontic therapeutic pain, such as the relevant factors causing dental pain, conduction mediators, and pain receptors [12]. At present, domestic and foreign scholars have started to study the mechanism of fixed orthodontic therapeutic pain at the molecular and cellular levels and found that therapeutic pain-related factors play an important role in both the peripheral and central mechanisms of fixed orthodontic pain. Since there are no specific pain receptors in the enamel, there is no pain sensation during orthodontic treatment, while the pulp and dentin contain many tiny nerve fibers, which contain mainly C-fibers and A-*δ* fibers [13]. The hypothesis proposed that any sensory nerve endings could produce some signals to conduct pain that was later given theoretical support [14].

The article "The Factors Affecting Orthodontic Pain with Periodontitis" was retracted in 2023. Reasons: suspected computer-generated content; unreliable results or conclusions; lack of ethics approval or compliance; missing or withdrawn patient consent.

It has been demonstrated that under orthodontic forces, the peripheral tissues contain small bundles of nerve fibers (C-fibers and A-delta fibers) that transmit information about the pain state to the nucleus of the pulpal ridge, some of which are dedicated to the transmission of pain signals and some of which are responsible for the transmission of both pain and general sensory signals. The pulp and periodontal tissues contain a large number of small nerve fiber bundles, mainly C-fibers and A-delta fibers, which are insulated and have a much faster conduction speed (10–30 m/s) than C-fibers (2.5 m/s), which are not insulated [15]. As the A-delta fibers (10–30 m/s) conduct faster, the pain sensation is mainly sharp, so the first sharp pain is perceived at the beginning of the first force application, and the C nerve fibers start to produce signals only after the sharp pain, resulting in a dull pain that is subjectively described as a “burning sensation”. The nerve fibers of the C nerve begin to produce signals only after the first sharp pain has been applied, producing a dull pain that the body subjectively describes as a “burning sensation” [16].

Burstone divided orthodontic pain into early pain and delayed pain. Early pain often occurs after the application of orthodontic forces, causing changes in the osmotic pressure in the periodontium; delayed pain is an allergic state of the periodontium, probably related to the stimulation of the nerve endings of the periodontium by inflammatory mediators, which in turn stimulates the release of neuropeptides from the pain receptors, usually within a few hours after the force is applied. It usually occurs within a few hours after the force is applied [17]. Recent studies have found that the effect and role of neuropeptides in the expression of orthodontic treatment of pain focus on neurokinin A (NKA), substance P (SP), neuropeptide Y (NPY), and calcitonin gene-related peptide CGRP.

The pain produced after the first force of a fixed orthodontic appliance does not only depend on the sensitization state of the periodontal membrane and the change in osmotic pressure caused by the stimulation but is also related to many factors, such as tooth separation, the value of the orthodontic force given, and other medical factors, as well as the sex and age of the individual, the variability of pain thresholds, and the psychological quality of the individual. In short, orthodontic pain after the first force is influenced not only by medical factors but also by psychological factors such as concentration, emotion, and the expected effect. Orthopedic pain after the first force is a series of reactions, both psychological and physiological, triggered by the action of a harmful stimulus on the body [18].

The article "The Factors Affecting Orthodontic Pain with Periodontitis" was retracted in 2023. Reasons: suspected computer-generated content; unreliable results or conclusions; lack of ethics approval or compliance; missing or withdrawn patient consent.

Therefore, how to relieve the pain caused by orthodontic treatment becomes the first consideration and problem for patients and practitioners [19]. At present, the commonly used methods to relieve orthodontic pain are reduction of orthodontic force, transcutaneous electrical nerve stimulation, oral analgesics, and certain low-dose laser irradiation [20]. The orthodontic force needs to reach a certain threshold in order to produce tooth movement, so it is impossible to reduce the orthodontic force indefinitely; oral analgesics have certain adverse effects, and it has been reported that analgesics also slow down the rate of movement of the malocclusion teeth and induce certain physical diseases; laser irradiation with a certain low dose must be operated by the physician and the pain relief has a certain time limit [21].

## 3. Introduction and Survey of Patients with Periodontal Disease

### 3.1. Clinical Information

One hundred patients with periodontal disease from October 2020 to May 2021 were treated with fixed orthodontic appliances and given orthodontic pain questionnaires. 11 invalid questionnaires were excluded (including those whose parents or patients did not complete the questionnaire, those who did not chew gum regularly as required, and those whose *L* factor *T* value in the Eysenck Personality Questionnaire was >60, i.e., highly masked and poorly credited). The remaining valid questionnaires were 89, with an effective rate of 89%. As shown in Figure 1, the pain transmission of the signals could be started to study the mechanism of fixed orthodontic therapeutic pain at the molecular and cellular levels and found that therapeutic pain-related factors play an important role in both the peripheral and central mechanisms of fixed orthodontic pain. There were 44 patients in the observation group, 18 males and 26 females; 34 were minors and 10 were adults. In the control group, there were 45 patients, including 19 males and 26 females; 34 were minor patients and 11 were adult patients.

The article "The Factors Affecting Orthodontic Pain with Periodontitis" was retracted in 2023. Reasons: suspected computer-generated content; unreliable results or conclusions; lack of ethics approval or compliance; missing or withdrawn patient consent.

Inclusion criteria for study subjects are as follows:

1. Patients with bimaxillary orthodontic treatment using straight wire orthodontic appliances
2. Both use Japanese TOMY straight wire arch brackets
3. Uniform use of Green Arrow chewing gum
4. Those who agree to participate in the survey and voluntarily fill out the questionnaire

Exclusion criteria are as follows:

1. Those with auxiliary devices such as bevel guides and implant supports in the oral cavity
2. Those with obvious endodontic and periodontal diseases
3. Pain caused by surgical procedures for maxillofacial deformities and oral soft tissue injuries caused by the interaction between brackets and bands
4. In addition to the observation group, patients in the control group who had chewing gum behavior during the experiment
5. Those who took antianxiety, analgesic, or sedative medication 4 days before wearing the aligner

## 4. Materials and Devices

The Short Form Mc Gill Pain Questionnaire (SF-MPQ) is a simplified version of the McGill Pain Questionnaire (MPQ), which was developed by Melzack and Torgerson in the 1970s to assess the intensity, characteristics, nature, and concomitant status of pain, and is one of the multifactor scoring methods for investigating pain. However, the content was cumbersome, abstract, and difficult to understand, so a simple, sensitive, and reliable pain assessment method, the Simplified McGill Pain Questionnaire (SF-MPQ), was proposed. The commonly used SF-MPQ includes pain index rating (PRI), pain intensity rating (PPI), and visual analog rating (VAS), among which the visual analog rating (VAS) is sensitive and reliable and is commonly used to assess dental pain in clinical practice, with the following steps: a line segment of about 100 mm long, 0 mm, and 100 mm is marked on both sides of the end. 0 mm is described as no pain and 100 mm is described as unbearable severe pain. 100 mm is described as intolerable severe pain. Between 0 mm and 100 mm, the tooth pain gradually increases and can be expressed as “soreness, swelling pain, mild pain, swelling pain, severe pain”. The point of the patient's tooth pain is marked on this line segment. This patient pain intensity rating value is the distance from 0 to this point. This method of assessing pain is simple, easy to understand, and highly feasible to operate.

The Eysenck Personality Questionnaire (EPQ) was developed by Professor H. J. Eysenck, a famous British psychologist, and the current version is available in two formats for children (7–15 years old) and adults (16 years old and above), covering a total of four parts respectively: *E* scale: measuring internal and external tendencies of personality; *N* scale: measuring emotional stability or neuroticism; *P* scale: measuring mental quality; *L* scale: testing the authenticity of the subject. This questionnaire has the advantages of being easy to understand and easy to test and having high validity and is one of the most influential psychological scales in the fields of psychology, medicine, education, and justice.

The article "The Factors Affecting Orthodontic Pain with Periodontitis" was retracted in 2023. Reasons: suspected computer-generated content; unreliable results or conclusions; lack of ethics approval or compliance; missing or withdrawn patient consent.

Psychotherapy and psychological interventions were first applied in the field of medicine by the famous psychologist Sigmund Freud in the 1920s, when he proposed the theory of “conscious and unconscious influence on their behavior”. The concept of psychological intervention is the process of using theoretical knowledge of psychology to systematically influence the psychological factors and personality traits of a given subject to bring about a change in their behavior toward the desired goal. Dental pain is the most common complication of orthodontic treatment; the main step in the implementation of psychological intervention in the treatment process is to inform the patient in detail of each step in the treatment process, the cooperation he needs to make, and the possible problems and solutions to problems, so that he can relax, eliminate his anxiety and panic, and reduce or eliminate the possible pain in the orthodontic process, so that he can better cooperate with the treatment. The treatment will be carried out in the following way.

The following methods of psychological interventions are commonly used in current clinical studies:

1. Psychological interventions for distraction.
2. Group-based psychological interventions.
3. Educational psychological interventions.
4. Cognitive a behavioral psychological intervention, etc. This study proposes using the distraction method; the so-called distraction is to shift their attention through some behavioral methods.

It has been reported in the literature that chewing gum can make people feel relaxed and in a more relaxed state physically and mentally, diverting the attention of patients from the pain caused by the orthodontic appliance and also better cooperating with the treatment. Therefore, this study used the chewing gum method, which has the advantages of easy implementation, low cost, safety, no side effects, good taste, and clean mouth.

## 5. Test Method

### 5.1. Investigation of Factors Influencing Pain

Before treatment, the orthodontist first made a record of some basic information of the patients and eliminated the samples that did not fit the requirements of this study. Patients who met the requirements of this experiment and participated voluntarily were given EPQ assessment questionnaires and tested by the physician. The patients were then randomly divided into two groups according to the order of consultation: the control group (conventional treatment mode) and the observation group (psychological intervention on top of the conventional treatment mode).

The article "The Factors Affecting Orthodontic Pain with Periodontitis" was retracted in 2023. Reasons: suspected computer-generated content; unreliable results or conclusions; lack of ethics approval or compliance; missing or withdrawn patient consent.

The patients selected for treatment with fixed orthodontic appliances in this experiment were cases of malocclusion with mild (moderate) crowding of the teeth, and all patients were required to keep a notational model after the initial visit and to take photographs of the oral and maxillofacial surfaces, which were printed and perfected for preservation to verify and ensure that all cases met the requirements of this experiment. For patients included in this experiment to cement the brackets and bands of the aligners, the labial and buccal surfaces were the first acids etched for 40 seconds, the acid etchant was rinsed, the labial and buccal surfaces were chalky, blown dry, and insulated, the brackets and buccal tubes were cemented with a small cotton ball coated with 3M bonding agent, and a 0.012-inch titanium-nickel round wire was placed on the first archwire. All brackets were lightly ligated with 0.020 mm stainless steel ligature wire to ensure that the same force was released from the archwire, the end of the archwire was bent back at the end with a needle holder, individual teeth that were tilted or twisted very significantly were not forcibly ligated into the slot first, and a light force was taken to suspend the ligature to avoid excessive force on the teeth causing pain to the patient already interfered with this experiment.

After the patients finished the initial orthodontic sticky wear, the professional staff immediately communicated with the patients and parents in the control group, introducing the knowledge about the treatment plan, precautions, and the maintenance of oral hygiene during the treatment period after wearing in, to relieve the patients' anxiety or nervousness, and explaining to them the purpose and significance of this experiment. All participating patients fully understood the purpose of this clinical study, voluntarily participated in this research study, could fully understand the questionnaire, and could accurately and honestly answer the pain reflections caused by wearing their own orthodontic appliances. The questionnaire required the patients to record the changes in pain at home for 2 h, 6 h, 24 h, 48 h, 72 h, 96 h, and 7 d after wearing the orthoses. The visual analog scales (VASs) were used to measure the intensity of dental pain to quantify the patients' pain level for the orthodontic treatment. 0 cm is described as “no pain”, 10 cm is described as “unbearable severe pain”, and between 0 cm and 10 cm, the pain increases gradually and can be described as “soreness, swelling, mild pain”. Patients marked the point on the line where the patient's tooth pain level was indicated, and the pain intensity was rated as the distance from 0 to that point. This questionnaire is to be filled out by the patient according to the preset time points and can be taken home. If there are minor patients, they can be supervised by their parents to complete this test together to ensure that no items are missed. Please bring the questionnaire with you when you return to the clinic so that it can be collected.

The article "The Factors Affecting Orthodontic Pain with Periodontitis" was retracted in 2023. Reasons: suspected computer-generated content; unreliable results or conclusions; lack of ethics approval or compliance; missing or withdrawn patient consent.

### 5.2. Introduction to Statistical Methods

The orthodontists involved in this experiment were all orthodontists with rich clinical experience, who fully understood the pain questionnaire and the Eysenck Personality Questionnaire, and were able to explain the issues related to the questionnaire carefully and accurately. Under the premise of establishing a good doctor-patient relationship, all patients should participate voluntarily and understand the purpose of the experiment and its clinical and scientific significance and have no interest in the relationship with themselves. All participating doctors should remind them to fill in the survey form and chew gum on time by telephone follow-up, respectively, and keep the test results confidential to protect patients' privacy, eliminate the subjects' concerns and worries, and ensure the authenticity of the test results. The physician regularly reminded all the participating patients by telephone to fill in the questionnaire form and chew the gum on time, as shown in Figure 2. In the curing satisfaction, pain contains not only pathophysiological factors and sensory effects but also multidimensional experiences, such as psychological factors, emotional effects, and individual subjective factors in the pain experience and the individual's unique experience. The measurement scores and data entry were done by one person, and another person was allowed to verify them.

After the questionnaires were returned, the same physician used the same ruler to measure the length of the pain point marked by the patient on the VAS from the 0 cm end:

1. Use of SPASS 11.0 (WINDOWS version) statistical software
2. Measures are expressed as mean ± standard deviation (*x* ± *s*)
3. One-way ANOVA was used between groups, and the significance level was set at *α* = 0.05, with *P* < 0.05 as a significant difference

## 6. Experimental Results

### 6.1. Influence of Gender and Age Factors

Some scholars have found that the pain caused by the first orthodontic force is more pronounced in female patients than in male patients, while others have found that there is no significant gender difference. In terms of sensitivity to dental pain caused by orthodontic treatment after the first force, it is generally believed that there are gender differences in orthodontic pain mainly due to the following considerations: first, there are three essential differences in the physiological structure of men and women, namely, differences in the reproductive system, differences in the occurrence of changes in hormone levels, and differences in hormonal composition; second, there are also differences in the function and structure of sympathetic nerve tissue between men and women; third, it is influenced by the social and psychological factors. The experimental group lies in asking patients to chew gum (uniformly Green Arrow gum) regularly after the initial orthodontic appliances. The professional staff issued orthodontic pain questionnaires to the patients and then explained to the patients and their families the method of filling them out so that they could fill out the questionnaires accurately, timely, and without errors:

1. Different upbringing, living environment, and social experiences make men and women express pain differently
2. Men and women have different levels of sensitivity to pain for physiological reasons
3. Differences in sociooccupational status of men and women result in different types of pain and different risks
4. Men and women have had different experiences of pain in the past

In this study, there was no significant difference in pain between the control group and the test group by gender (*P* > 0.05). The reason why this result is inconsistent with the results of previous studies may be that although women are prone to anxiety and fear of pain in many cases, they have a high demand for beauty and are also very tolerant. Therefore, women's requirements for appearance and their awareness and acceptance of orthodontics may lower their pain threshold. In this study, due to time, manpower, and financial constraints, the sample content selected for this study was small and the observation time of the patients was relatively short, and in future work, it will be necessary for the latter to increase the information of large samples for further study. The pattern of influence of sociodemographic factors between the control and observation groups is as follows. The sociodemographic factors of the control and observation groups were compared, and no statistically significant differences were found between the two groups in terms of gender (*P*=0.412) and age (*P*=0.723) (as shown in Figure 3).

The article "The Factors Affecting Orthodontic Pain with Periodontitis" was retracted in 2023. Reasons: suspected computer-generated content; unreliable results or conclusions; lack of ethics approval or compliance; missing or withdrawn patient consent.

The basic pattern: no pain was felt; pain developed and gradually increased (the onset of tooth pain ranged from 1 h to 11 h, with an average time of 2 h) in 89 patients with the exception of 3 patients who did not experience pain. Reaching the peak (around 24 h), the pain gradually decreases, and then, there is no pain (see Figure 4) (pain scores at different time points in both groups of patients).

### 6.2. Factors Influencing Tooth Pain after Stressing with Meals

Comparing the pain values in one week between the two groups of patients of both sexes, the difference was not statistically significant (*P* > 0.05), which shows that dental pain is not related to gender. Comparing the pain values within one week between the two groups of patients of age, the difference was statistically significant (*P* < 0.05), which shows that dental pain is related to age (see Figure 5).

The International Society for the Study of Pain has standardized the definition of pain as follows: “pain is an unpleasant sensory and emotional sensation associated with substantial or underlying tissue damage”. In this definition, pain contains not only pathophysiological factors and sensory effects but also multidimensional experiences, such as psychological factors, emotional effects, and individual subjective factors in the pain experience and the individual's unique experience. Pain as a subjective experience varies greatly among individuals, as evidenced by their perception and tolerance of pain, and orthopedic pain is also influenced by the patient's mental attention, emotions, pain experience, and genetics, making it difficult to evaluate. In psychology, the visual analog scale (VAS) was the first to quantify emotion as a method of evaluating acute and chronic pain, and its sensitivity is outstanding. Therefore, the visual analog scale was chosen to assess orthopedic pain in this experiment.

The Eysenck Personality Questionnaire (EPQ) is one of the most influential psychological scales in the fields of psychology, medicine, education, and justice because it is easy to understand, is simple to administer, and has high validity. The EPQ questionnaire consists of yes or no questions, and after the test is completed, the total score is calculated and converted into a standard score, where *L* is a validity scale, and if *L* > 60, the patient has strong masking information and is excluded. Since this experiment is a multifactor questionnaire, this study was conducted by testing the balance of sociodemographic factors between the control group and the experimental group, which to some extent reduces the unfavorable factors affecting the accuracy of this study and avoids research bias.

### 6.3. Influence of Psychological Factors

The pain levels of the observation group and the control group were different at different time points, the pain value of the control group was greater than that of the observation group at each time point, the difference was statistically significant (*P* < 0.05), and the specific scores of pain are shown in Figure 6. However, the trend of pain time change was basically the same in both groups, and the pain started to appear at about 2 h, and then, the pain time was gradually prolonged and the pain gradually increased until the pain level at 24 h. The intensity of pain gradually decreased until it disappeared completely on the seventh day.

The article "The Factors Affecting Orthodontic Pain with Periodontitis" was retracted in 2023. Reasons: suspected computer-generated content; unreliable results or conclusions; lack of ethics approval or compliance; missing or withdrawn patient consent.

Orthodontic pain is chronic pain with a short period, low intensity, and obvious individual differences. 90% to 95% of orthodontic patients have experienced varying degrees of pain or discomfort during the orthodontic treatment process. The study showed that, at the beginning of the first force of the fixed orthodontic treatment, up to 94% of the population felt varying degrees of tooth pain, which usually manifested itself as tooth pain and discomfort in 2–3 h after the force was applied to the orthodontic patient, with the tooth pain peaking in 1–2 d. Then, the pain gradually disappeared in 3–7 d. The majority of orthodontic patients basically felt no pain on the 7th day. In this experiment, 2 h, 6 h, 24 h, 48 h, 72 h, 96 h, and 7 d after the initial orthodontic braces were selected as the observation time, mainly because the pain-related factors and pain mediators and pain receptors will change differently over time at these different time points of orthodontic therapeutic pain. A questionnaire was administered to the patients to obtain clinical information about their perceived pain after wearing orthodontic appliances. After data processing and statistical analysis, it was found that 3 of the 89 patients who wore straight wire orthodontic appliances with valid questionnaires complained of no pain, while the remaining patients complained of pain of varying degrees from 1 h to 11 h, with the average time of pain perception being more than 2 h, with the peak of pain perception occurring approximately 24 h after wearing the appliances, followed by a gradual decrease in pain by the seventh day. The majority of patients complained of no more pain, as shown in Figure 7. The results of this experiment are generally similar to those reported in the literature above. Now, it has been confirmed that this pain pattern affects the synthesis and secretion of neural factors, and the orthodontic therapeutic pain pattern is as follows: no pain felt, pain generated and gradually increased, peaked, the pain gradually decreased, and no pain. The pain gradually decreases and no pain.

The article "The Factors Affecting Orthodontic Pain with Periodontitis" was retracted in 2023. Reasons: suspected computer-generated content; unreliable results or conclusions; lack of ethics approval or compliance; missing or withdrawn patient consent.

The mechanisms involved, according to available literature and experimental reports, are probably:

1. After wearing the orthodontic appliance, the tensioned fibers on the tensioned side of the tooth impact the peripheral nerve fiber endings and the nerve endings of the periodontal membrane and fail to conduct the pain sensation, which is restored after about 2 hours.
2. Wearing the orthodontic appliance may cause temporary local ischemia or aseptic necrosis, resulting in a decrease in the threshold of pain perception and an increase in pain after about 1 day, and then, with the extension of wearing time and completion of tooth movement, the actual force exerted by the orthodontic appliance on the teeth decreases, the pain receptors of the teeth and periodontium regain their function, and the pain threshold rises and approaches the original level, but the receptors fully regain their ability to discriminate between painful stimuli. The ability to discriminate between painful stimuli requires the end of orthodontic treatment to be reached.
3. The periodontal ligament is stretched to release some chemical mediators, which are distributed in different concentrations in the periodontal membrane at different times, producing different painful stimuli.
4. The pain produced by the force exerted on the teeth after wearing the orthodontic appliance is divided into immediate pain and delayed pain depending on the time of generation. Immediate pain may be related to the pressure response to the periodontal ligament caused by the force exerted after wearing the orthodontic appliance; delayed pain may be due to the periodontal membrane nerve fiber endings being in a hypersensitive state, often produced several hours after the first force is exerted. The occurrence of delayed pain is mainly related to the chemical mediators produced by the nerve endings in the periodontium after stimulation by force and the neuropeptides released by the periodontal pain receptors after stimulation by orthodontic force.

### 6.4. Factors Influencing Pain during Treatment

With the awareness that patients with malocclusion are primarily interested in the aesthetics of their teeth, there is a significant difference in the response of adult and adolescent patients to orthodontic pain. Medical experts also have different opinions regarding the age-related differences in therapeutic pain and the age-related differences in tooth pain caused by the first force applied to orthodontic treatment. The theoretical basis for these opinions may be the fact that adolescent patients are more likely than adults to experience pain after the first force, probably because adolescents are not yet psychologically developed and are prone to psychological discomfort from orthodontic pain; on the other hand, it may be that adolescent patients' newly erupted teeth are young permanent teeth and their dental and periodontal tissues are not yet mature, so they are more active in the tissue alterations caused by orthodontic force. On the other hand, it may be due to the fact that the periodontal and periodontal tissues of the young permanent teeth have not yet developed and are not mature enough for the tissue alteration caused by the orthodontic force, or that there is a difference in the level of perceptual threshold of periodontal and pulpal tissues to the tooth pain caused by the force in different age groups, or that the psychological tolerance of different age groups is different. In this experiment, there was a significant difference (*P* < 0.05) in the pain level between the two groups of patients of different ages, as shown in Figure 8, where the pain level of adult patients was higher than that of adolescent patients. This may be due to the fact that although adult patients have mature dental pulp and periodontal tissues and are in a social environment with better compliance and self-control than adolescents, they show more concern about the treatment course, efficacy, and possible risks of the whole orthodontic treatment process, repeatedly consult the doctor about everything, and sometimes lack trust in the doctor and are under great psychological pressure, which leads to the perception of pain by periodontal tissues and dental pulp. This leads to a lower threshold of pain perception in the periodontal tissues and dental pulp and thus a stronger sensitivity to pain than in adolescents. The pain caused by the first orthodontic force contains not only pathophysiological factors and sensory effects but also multidimensional experiences, such as psychological factors, emotional effects, individual subjective factors, and unique experiences in the pain experience. Recent research data suggest that the psychological fluctuations caused by tooth movement after force may precede the pain sensation induced by the pain receptors and that the psychological stress experienced by the patient during the treatment may also have an impact on the pain perception. Chewing gum can distract patients and is one of the methods of psychological intervention. In this experiment, the chewing gum method was used to test the effect of psychological factors on pain, and from the comparison of the control and experimental groups, it was seen that chewing gum significantly reduced the level of pain that occurs during orthodontic treatment. Therefore, psychological factors are one of the most important factors influencing dental pain after orthodontic stress.

The article "The Factors Affecting Orthodontic Pain with Periodontitis" was retracted in 2023. Reasons: suspected computer-generated content; unreliable results or conclusions; lack of ethics approval or compliance; missing or withdrawn patient consent.

The results of this experiment showed that the pain pattern using chewing gum changed in the same trend as the control group and was not statistically significant, but this psychological intervention method was able to reduce the intensity of orthodontic therapeutic pain. Therefore, chewing gum did not change the essence of the process of perceived pain and the basic pattern of occurrence and progression of pain in patients after the first force of the initial orthodontic appliance, but it could alleviate the degree of pain. The reasons for this may be the following:

1. Chewing gum can make people feel relaxed and in a more relaxed state physically and mentally, diverting the patient's attention from the pain caused by the orthodontic appliance and also better cooperating with the treatment
2. Chewing gum can accelerate the blood circulation inside and outside the periodontal membrane, promote periodontal lymphatic circulation, further reduce and prevent the production of inflammatory chemical mediators and neuropeptides, and reduce the occurrence of tissue edema
3. Chewing gum to accelerate blood flow can also block the transmission of pain signals via nerve impulses to relieve pain

## 7. Conclusion

The purpose of the paper was to investigate the basic patterns and influencing factors of dental pain in fixed orthodontic patients within seven days after the initial wearing of straight arch aligners and the analysis of the effect of psychological intervention on dental pain using the visual simulation scoring method. According to the inclusion criteria of the experimental design, 89 patients who visited the Department of Orthodontics of Hospital for malocclusion were randomly divided into observation group and control group, and the observation group used chewing gum as psychological intervention, while the control group did not use any intervention. The effect of psychological intervention on periodontal pain was analyzed. The results of the paper were that all but 3 of the 89 patients had no pain, and all the patients had different degrees of dental pain at different points in time. Dental pain was related to age, *P* < 0.05, and the difference was statistically significant; it was not related to gender, *P* > 0.05, and the difference was not statistically significant. The trend of pain change was the same in the observation and control groups, and the control group was greater than the observation group at all time points, *P* < 0.05; the difference was statistically significant.

## Figures and Tables

**Figure 1:** Pain transmission in periodontal disease.

The article "The Factors Affecting Orthodontic Pain with Periodontitis" was retracted in 2023. Reasons: suspected computer-generated content; unreliable results or conclusions; lack of ethics approval or compliance; missing or withdrawn patient consent.

**Figure 2:** Examination procedure for patients with periodontal disease.

**Figure 3:** Comparison of sociodemographic factors between the two groups of patients.

**Figure 4:** Pain scores at different time points for both groups of patients. (a) Experimental group. (b) Blank group.

**Figure 5:** Changes in pain index by gender and age.

**Figure 6:** Effect of fear on pain rating.

**Figure 7:** Cycle of pain change. (a) The first cycle. (b) The second cycle. (c) The third cycle.

**Figure 8:** Pain levels in patients of different ages.

## Data Availability

The data used to support the findings of this study are available from the corresponding author upon request.
